RETRACTED

# A Composite Particle Swarm Optimization Algorithm for Hospital Equipment Management Risk Control Optimization and Prediction

**DOI:** 10.1155/2022/5268887

**Published:** 2022-05-23

**Authors:** Jinghui Li, Li Zhang, Xiangmin Gu

**Affiliations:** ^1^Department of Hospital Office, Jiangsu Taizhou People's Hospital, Taizhou 225300, China; ^2^School of Politics and Public Administration, Shanxi University, Taiyuan 030000, China; ^3^Immunization Program Division,Tianjin Binhai New Area Disease Prevention and Control Center, Tianjin 300270, China

## Abstract

Aiming at the problem that particles cannot realize multidimensional analysis and poor global search ability, a composite particle swarm optimization algorithm is proposed, improving the accuracy of particle swarm optimization. Firstly, k-clustering is used to cluster risk management particle swarm optimization. The advantages of particle swarm optimization have to be given full play, and the risk of hospital equipment management from various aspects has to be controlled. Then, the multidimensional particle swarm is segmented to obtain an ordered multidimensional risk particle swarm set, which provides a basis for later risk prediction. Finally, through the fusion function of multidimensional risk particle swarm, the risk particle swarm set based on the clustering degree is constructed, and the optimal extreme value is obtained, so as to improve the accuracy of management risk calculation results. Through MATLAB simulation analysis, it can be seen that the composite particle swarm optimization algorithm is better than particle swarm optimization algorithm in global search accuracy and search time. Moreover, the calculation time and accuracy are better. Therefore, the composite particle swarm optimization algorithm can be used to analyze the risk of hospital equipment and effectively control the risk of hospital equipment management.

## 1. Introduction

In recent years, the state has strengthened the management of medical equipment and made medical sector pay more attention to the control of equipment management risk. Hospital equipment is the basis of medical work and plays an important role in treatment effect. There are many influencing factors of hospital equipment management risk [1], most of which are unstructured qualitative factors, and the relationship between each factor and management risk is nonlinear, so risk analysis is difficult. Some scholars believe that clustering function can effectively improve the level of hospital equipment management and reduce the incidence of related risks. At the same time, the clustering function can make up for the shortcomings of the particle swarm optimization algorithm, improve the local search ability, analyze the results more accurately, and predict the future development trend [2]. The combination of k-cluster analysis and the particle swarm optimization algorithm can realize the joint optimal result analysis and make each index more accurate. It is a comprehensive analysis method. After integrating the k-clustering algorithm, the self-learning mechanism of the algorithm can be improved, clustering and subcontracting problems can become clearer, and the massive data analysis of hospital equipment management can be realized. Hospital equipment management is an important asset. If the management risk cannot be predicted in advance, it will increase the incidence of medical accidents and the loss of state-owned assets. It is an urgent problem to find an objective and accurate equipment risk control method. The composite particle algorithm will be able to perform comprehensive analysis of hospital equipment, risk control from various aspects, and multiangle research, making the results more accurate. The composite particle algorithm makes up for the shortcomings of the particle algorithm, further exerts the iterative advantages of the particle algorithm, and simplifies the calculation process. The fusion of the K-clustering algorithm and particle algorithm can simplify the number of particles and realize massive data analysis and is suitable for a large number of hospital equipment analysis and risk prediction. Therefore, the integration of cluster analysis and the particle swarm optimization algorithm can comprehensively analyze the influencing factors in hospital equipment management, better predict the corresponding risks, and facilitate the management of hospital equipment. Some scholars have fused the particle swarm optimization algorithm with Bayesian theory and found that the joint analysis method can improve the effectiveness of hospital equipment management and enhance the ability of risk management. The combination of cluster analysis and the particle swarm optimization algorithm can comprehensively analyze the influencing factors in hospital equipment management, better predict the corresponding risks, and facilitate the management of hospital equipment. Some scholars combine the particle swarm optimization algorithm with Bayesian theory and find that the joint analysis method can improve the effectiveness of hospital equipment management and enhance the ability of risk management [3]. Some scholars verify the fusion of particle swarm optimization and the neural network through actual case analysis and find that its calculation result is better than a single particle swarm optimization algorithm [4]. Other scholars conducted multifactor regression analysis for hospital equipment management and found that the particle swarm optimization algorithm has the problem of high discreteness, which will reduce the accuracy of calculation results [5]. Based on the above background, this paper makes a quantitative analysis of the relevant parameters in hospital equipment management, comprehensively analyzes the fusion between k-clustering and the particle swarm optimization algorithm, and verifies the effectiveness of the algorithm.

RETRACTED

## 2. Overview of Relevant Parameters

### 2.1. Particle Swarm Optimization

Particle swarm optimization is a comprehensive statistical stochastic method, which mainly uses the randomness analysis of particles to solve systematic problems [6], and is widely used in various fields. The particle swarm optimization algorithm uses continuous analysis and utilizes the occurrence probability of different particles to search the final result. The particle swarm optimization algorithm first searches for the global optimal solution and then searches for the local optimal solution [7]. Suppose 1: *g*_*it*_ is a multidimensional collection of particles, where the dimension of *i* particle, the position of *t* particle, and *x* is any particle. Suppose, *P*_*j*_(*x*)=∑_*i*,*t*=1_^*n*^{*g*_*it*_^*j*^*·k|g*}, *k* ∈ (1, ⋯*n*), then *P*_*j*_(*x*) is the global optimal position of the particle *g*_*it*_. Because the randomness of the particle swarm is normal, the global optimal position of particles is fluctuating, which is *g*_*it*_=2  sin(tan  *πt*/*ρ*), when the global position of the particle swarm is optimal, where, *ρ* is the minimum prime set, and 2  sin  (tan  *πt*/*ρ*)^*j*^*·k* < ∑_*i*,*j*,*t*=1_^*n*^{*x*_*it*_^*j*^*·k*}.

**Theorem 1 .**

The calculation function of *P*_*n*_(*x*) the local optimal position is *f*(·) ∈ *B*_*t*_ (the eigenvalue of *B*_*t*_ the *t* position); then the calculation formula of the overall optimal position is

(1) $$\begin{array}{c} \int_{x\in g_{ij}}f\left(x\right)dx-\bar{\sum_{j=1}^{n}f\left(P_{j}\left(x\right)\right)}<\hat{Q}\left(f\left(x\right)\right), \end{array}$$

where the function is *Q*(*f*(*x*)) calculated for the eigenvalue of *f*(·).

**Theorem 2 .**

Different derivatives *f*(*x*) satisfy the following conditions, *f*(*x*) < max(*x*), *f*(*x*)′ < max(*x*)′…., *f*(*x*)^*j*^ < max(*x*)^*j*^, then all local eigenvalues are within *f*(*x*)′, and the error is less than*lin*(*x*)′.

**Theorem 3 .**

Any point *x*_*it*_ in the particle swarm is randomly distributed in the multidimensional space, and the deviation of any point is*D*(*x*). The calculation formula is as follows:

(2) Dx,fx=limx⟶∞x·logPjxt,

where *D*(*x*, *f*(*x*)) is the projection of deviation between [0, 1].

RETRACTED

According to the above theorem, the relationship between the change amplitude and the amount of data *x* can be obtained by approximate integration [8], which is independent of the spatial dimension *i*. Therefore, deviation projection analysis of particle swarm optimization provides a good theoretical basis for multidimensional particle swarm analysis. According to Theorem 3, the uniform deviation linx·logPjxt between the particles can effectively control the variation amplitude. Some scholars combine the particle swarm optimization algorithm with wavelet function to propose the composite particle swarm optimization algorithm. It is proved that the ability of the algorithm to control the data amplitude is consistent with the analytical conclusion proposed in this paper [9]. Therefore, this paper transforms the particle swarm optimization data to realize multidimensional analysis.

### 2.2. The Clustering Function

*K*-clustering function is used for particle swarm optimization, Euclidean distance is used to divide clustering degree, and self-learning is carried out through self-adaptability [10], constantly revising the relationship between the clustering sets. K-clustering uses “IF” to judge ranking between different clusters, and different clustering results are obtained under the Euclidean distance *S* as follows.

IF: *x*_*i*_ ∈ *g*_*ij*_ and *S*(*x*)=max(*x*_*i*_, *x*_*j*_), *x*_*i*_ and *x*_*j*_ are the two boundary points of clustering, respectively, then $S=\bar{\sum_{i=1}^{n}s\left(x_{i}\right)\cdot k/q}$,

where *k* is the weight coefficient of particles, *g*_*ij*_ is the particle set, *S*(*x*) is the Euclidean distance, and max(*x*_*i*_, *x*_*j*_) is the maximum value of the Euclidean distance. K-clustering can analyze unstructured and structured data, process through different Euclidean distances, output clear results, and obtain the optimal combination of complex data structures [11].

**Hypothesis 2 .**

rbitrary particles *x*_*i*_, after sorting by the Euclidean distance *S*, the clustering relationship between the input variables *x*_*i*_ and output variables *y*_*i*_ can be obtained, as shown in (3).

(3) $$\begin{array}{c} g_{ij}=\sum_{i,j=1}^{n}g\;\exp\left\{\frac{\left(x_{i}-x_{j}\right)}{q}\right\}, \end{array}$$

where *q* is the cluster center; exp*()* is the expected function, and *g*_*ij*_ is the cluster set.

By performing k-clustering calculation on the above expected functions, the continuous operator of k-clustering can be obtained, as showed in (4).

(4) $$\begin{array}{c} g_{ij}=k\cdot \overset{⟶}{\sum_{i,j,k=1}^{n}g_{ij}^{t}\left(x\right)}, \end{array}$$

where *k* is the clustering coefficient, and *t* is the derivation coefficient. According to clustering, the output value is obtained:

(5) $$\begin{array}{c} y=k\cdot \frac{\left[\sum_{i,j=1}^{n}\overset{⌢}{g_{ij}^{i}\left(x\right)\cdot f\left(P_{j}\left(x\right)\right.}\right]}{\max\sum_{i,j=1}^{n}g_{ij}^{i}\left(x\right)}. \end{array}$$

K-clustering not only reduces the amount of data processing, but also realizes the orderly analysis of data through the Euclidean distance. At the same time, k-clustering reduces the influence of dimension on the results after multiple derivations Pramanik et al. [12], realizes the multidimensional calculation of particle swarm optimization, and improves the accuracy of calculation.

RETRACTED

## 3. Build the Risk Control Model of Hospital Equipment Management Based on the Complex Particle Swarm Optimization Algorithm

### 3.1. The Convolution of Initial Data

The risk control model of hospital equipment management constructed in this paper needs to realize accurate complex data calculation and improve the search ability of characteristic data, so it needs multidimensional coevolution. The model uses the convergence threshold and k-clustering factor to realize the convolution of distributed particle swarm optimization and obtain the eigenvalue of the best variation range [13].

(1) Initialization of particle swarm. The particle swarm optimization algorithm believes that the initial particles are randomly distributed, there is a strong uncertainty, and its calculation process is complex. The particle swarm optimization algorithm must be attracted by the relatively concentrated particle set. It will fall into local optimization and increase the error rate of calculation results. Therefore, improving the order of particles, reducing the influence of random particles on the calculation results, expanding the number of particle sets, and solving the local optimization problem are the key [14].
The k-clustering method can process particles in an orderly manner, changing the randomness of particles into the randomness of particle sets. The results are shown in Figures 1 and 2.
Figures 1 and 2 show the multidimensional initial swarm of the particle swarm optimization algorithm and composite particle swarm optimization, respectively, and the number of a swarm is 120. Through comparison, it is found that the arrangement of the particle swarm is more chaotic, and the composite particle swarm is more concentrated. Moreover, the data set constructed by the composite particle swarm optimization algorithm is independent of spatial dimension. The distribution effect of each point is the same, and data distribution is strong [15].
(2) Multistrategic collaboration. Multistrategy collaborative search is a progressive search of multiple strategies according to different k-clustering levels. In order to reduce the calculation time of particle swarm optimization, a multistrategy calculation method is adopted. At the same time, several common strategies of particle swarm optimization are analyzed as follows:
  (1) Self-progression
    (6) $$\begin{array}{c} y_{ij}\left(t+1\right)=k\cdot y_{ij}\left(t\right)+c_{1}\cdot \frac{\left[k\cdot \sum_{i,j,k=1}^{n}g_{ij}^{k}\left\{x\left(t\right)\cdot f\left(P_{j}\left[x\left(t\right)\right]\right.\right\}\right.}{\text{mean}\sum_{i,j=1}^{n}g_{ij}^{t}\left[x\left(t\right)\right]}. \end{array}$$
  (2) Global progressive
    (7) $$\begin{array}{c} y_{ij}\left(t+1\right)=k\cdot y_{ij}\left(t\right)+c_{2}\frac{\left[k\cdot \sum_{i,j=1}^{n}g_{ij}^{t}\left\{x\left(t\right)\cdot f\left(P_{j}\left[x\left(t\right)\right]\right.\right\}\right.}{\text{all}\sum_{i,j=1}^{n}g_{ij}^{t}\left[x\left(t\right)\right]}. \end{array}$$
  (3) Progressive structure
    (8) $$\begin{array}{c} y_{ij}\left(t+1\right)=k\cdot \left|\frac{\left[\delta \cdot \sum_{i,j=1}^{n}g_{ij}^{t}\left\{x\left(t\right)\cdot f\left(P_{j}\left[x\left(t\right)\right]\right.\right\}\right.}{B\left(\sum_{i,j=1}^{n}g_{ij}^{t}\left[x\left(t\right)\right]\right)}\right|, \end{array}$$
where *c*_1_ and *c*_2_ are the synergy coefficients of different strategies. *K* is the clustering degree of different strategies, *n* is the number of different strategies, *B ()* is a Boolean function, and *Lin ()* is a linear function. In this paper, universal particle swarm optimization has been improved in two aspects. On the one hand, the search range is expanded as much as possible, and a sequence is randomly selected from five forms for self-progression. *K*-clustering is utilized to randomly assign each particle swarm to increase the search accuracy of local optimal solution. On the other hand, the global convergence needs to be improved, and the calculation time is saved [16].
(3) Collaborative strategies in different dimensions. Composite particle swarm optimization adopts the/a differentiation strategy for particles with different dimensions and realizes multidimensional distributed collaboration by adjusting the corresponding parameters, so as to complete convolution. K-clustering clusters the particles with different dimensions to obtain different subparticle groups and uses multiple collaborative strategies for iterative calculation. Particle swarm optimization with different dimensions uses the fitness function to adjust dimensions and select strategies. The fitness function can be simplified and progressive, get the optimal value, and increase the speed and accuracy of the search.

RETRACTED

### 3.2. The Risk Controls the Method of Hospital Equipment Management Based on the Composite Particle Swarm Optimization Algorithm

The composite particle swarm optimization algorithm can realize dimensional coevolution and optimize the initial value, threshold and parameters of particle swarm optimization to obtain the optimal solution, and the shortest computing time [17].

The flow of the experiment is shown in Figure 3.

**Step 1 .**

Determine the dimension and data structure of particle swarm optimization and determine the data structure of the time series according to the data characteristics of hospital equipment management risk control. The initial weight and threshold of the whole data are considered as a whole to form different cluster sets. Each cluster set is arranged according to its dimension, weight, and threshold. According to the actual application, the time series dimension *g* *=* 350 is determined.

**Step 2 .**

Data initialization. Randomly initialize the relevant parameters of particle swarm optimization. Let the number of particle swarm *n* *=* 50, the maximum weight belongs to {0.2, 0.3}, and the maximum number of iterations *D* *=* 350.

**Step 3 .**

uild the appropriate function, using the k-clustering theory to generate initial sequences with different dimensions and according to the initial weight and threshold. Through the self-learning and training of (1) ∼ (7), the synergy coefficient is continuously improved to obtain the appropriate function.

**Step 4 .**

earch the global optimal position and the optimal position of each subtime series, randomly use the five strategies to obtain the fitness ratio, and record the global optimal position and the optimal position of each subseries.

**Step 5 .**

udge whether the maximum number of iterations has been reached. If it has been reached, the calculation will be switched off. Otherwise, repeat steps 2–6 to return the results such as threshold, weight, and the optimal position [18].

## 4. The Case Study on Risk Control of Hospital Equipment Management

### 4.1. Effectiveness Judgment of the Composite Particle Swarm Optimization Algorithm

The commonly used detection functions of particle swarm optimization, sphere, restoring, and Ackley are analyzed and compared with the particle swarm optimization algorithm to verify the accuracy of the results. The data for this study come from the statistical yearbook, and the reliability and validity of all questionnaires are greater than 0.7. Sphere detects the global search ability of the particle swarm optimization algorithm, and the formula is as follows:

(9) $$\begin{array}{c} f\left(x\right)=k\cdot \sum_{i=1}^{n}\hat{\left[x_{i}^{2}\right]}. \end{array}$$

The local extremum of restoring the detection function, the formula is as follows:

(10) $$\begin{array}{c} f\left(x\right)=\sum_{i=1}^{n}\left[x_{i}^{2}-\max\left[10\pi \left(2\pi x_{i}\right)\right]+\pi \right]. \end{array}$$

Ackley is a gradient optimization function of multidimensional points to test the calculation speed of multidimensional data to detect the global convergence speed. The formula is as follows:

(11) $$\begin{array}{c} f\left(x\right)=-20\;\exp\left\{-0.2\sum_{i=1}^{n}\sqrt{\hat{\sum_{i=1}^{n}x_{i}^{2}}}\right\}-\exp\left\{\hat{\sum_{i=1}^{n}\cos\left(2\pi x_{i}\right)}\right\}, \end{array}$$

where *n* is the number of samples, *x*_*j*_ is particle swarm optimization, and *x*_*i*_ is the risk management of any equipment. The value ranges of projection in each function are {−1, 1} [19].

RETRACTED

In order to facilitate calculation, the number of particle swarm in this paper is *n* = 50, the maximum algebra is *D* = 350 time, and the dimensions are 4 dimensions. Function tests of 3 dimensions are carried out, respectively. In order to ensure the accuracy of the results, the average multiple values of the results have to be taken. The specific calculation results are shown in Table 1.

It can be seen from Table 1 that the global optimal solution of the test function in 3 is 1, and the standard deviation and mean value meet the test requirements. In terms of the mean deviation and standard deviation, the calculation results of composite particle swarm optimization are better than those of the particle swarm optimization algorithm, indicating that the former is better. In order to further prove the results in Table 1, the test functions in 3 are analyzed, respectively, and the results are shown in Figures 4–6.

It can be seen from Figure 4 that the optimization range and error rate of the sphere function are decreasing, indicating that the sphere function inspection effect of the composite particle swarm optimization algorithm is good. However, convergence results of sphere function optimization show volatility, mainly from global search to local search.

It can be seen from Figure 5 that the optimization range and error rate of the restoring function are shrinking, indicating that the restoring function inspection effect of the composite particle swarm optimization algorithm is good, and the local search results are relatively stable.

It can be seen from Figure 6 that the optimization range and error rate of Ackley are shrinking, indicating that the search time of the Ackley function of the composite particle swarm optimization algorithm is short. At the same time, the function also shows volatility, which is also due to the shift from the global search to local search.

RETRACTED

### 4.2. Introductions to Risk Cases of Hospital Equipment Management and Control

This paper selects the medical equipment management control data from April 1, 2019, to April 1, 2021, as the sample to analyze the equipment management control risk. Equipment management includes intellectual property, management technology, management pictures, management audio, account number, supplier, and equipment damage. The risk assessment standard of the sample refers to the national medical equipment management measures, hospital medical equipment management specifications, and regional medical equipment management guidance schemes to judge the control risk of equipment management, which is divided into five levels: high-risk, medium risk, general risk, normal risk, and low-risk levels. In order to facilitate the analysis, the data from April 1, 2019, to April 1, 2020, are taken as the analytical data, and the data from April 1, 2020, to April 1, 2021, are taken as the prediction data for comparative analysis. Among them, the incomplete data are supplemented by the filter function of the particle swarm optimization algorithm, and the results are shown in Table 2.

### 4.3. The Test Results

In order to verify the effectiveness of the composite particle swarm optimization algorithm proposed in this paper, compared with the particle swarm optimization algorithm, the calculation accuracy and calculation time are shown in Figure 7.

As can be seen from Figure 7, the calculation time of the composite particle swarm optimization algorithm is less than that of the particle swarm optimization algorithm, which shows that the calculation efficiency of the composite particle swarm optimization algorithm is higher, and the time of the particle swarm optimization algorithm changes greatly. The calculation accuracy and time of both algorithms are shown in Table 3.

It can be seen from Table 3 that the calculation accuracy of the composite particle swarm optimization algorithm is greater than 95%, while the calculation accuracy of particle swarm optimization algorithm is about 90%. Therefore, accuracy of composite particle swarm optimization algorithm is better. The reason is that the composite particle swarm optimization algorithm adjusts the synergy coefficient, weight, and convergence factor through k-clustering to make the calculation result better.

## 5. Conclusion

In this paper, k-clustering and particle swarm optimization algorithm are combined to realize multidimensional coevolution of hospital equipment management risk [20]. At the same time, the threshold and weight of risk control are adjusted to obtain the control model of hospital equipment management risk. Comparing the composite particle swarm optimization algorithm with the particle swarm optimization algorithm, the results show that the composite particle swarm optimization algorithm has better prediction accuracy and convergence and can predict the risk of hospital equipment management. The calculation accuracy of the composite particle swarm optimization algorithm is greater than 95%, while the calculation accuracy of the particle swarm optimization algorithm is about 90%. However, in this model, the multidimensional collaborative strategy pays too much attention to the global search ability, resulting in the relative decline of the local search ability, and ignores the correlation between hospital equipment management risk indicators. Therefore, in the future research, the index adjustment coefficient will be added for improvement.

RETRACTED

## Figures and Tables

**Figure 1:** Particles processed by the composite particle swarm optimization algorithm.

**Figure 2:** Particles processed by the particle swarm optimization algorithm.

**Figure 3:** The risk control process of hospital equipment management based on the composite particle swarm optimization algorithm.

**Figure 4:** The convergence results of sphere function optimization.

**Figure 5:** The convergence results of restoring function optimization.

**Figure 6:** The optimization time of the Ackley function.

**Figure 7:** The variation range of calculation time of different algorithms.

**Table 1:** The test time and results of test function.

Detection function	Algorithm	Value range	Mean difference (E)	Standard deviation (E)	Global optimal solution
Sphere	Composite particle swarm optimization	1.31*E* − 6∼0.23*E* − 11	0.13–7	0.02–6	1
	Particle swarm optimization	1.22*E* − 7∼0.14*E* − 10	0.23–8	0.02–8	

Rastrigin	Composite particle swarm optimization	1.23*E* − 7∼1.03*E* − 11	0.02–7	0.01–8	1
	Particle swarm optimization	1.61*E* − 4∼1.43*E* − 10	0.03–4	0.01–5	

Ackley	Composite particle swarm optimization	1.42*E* − 7∼1.03*E* − 13	0.04–7	0.01–8	1
	Particle swarm optimization	2.12*E* − 6∼1.03*E* − 13	0.13–6	0.01–7	

**Table 2:** The equipment management risk classification results.

Risk level	Data volume (PCs.)	Proportion (*%*)
The high-risk level	1202	20.82
The medium risk level	432	7.48
The general risk level	2032	35.19
The normal level	1041	18.03
The low-risk level	1067	18.48

**Table 3:** The prediction accuracy and time at different levels.

Algorithm	Prediction accuracy of different risk levels (%)					Calculation time (seconds)
	The high-risk level	The medium risk level	The general risk level	The normal level	The low-risk level	
Composite particle swarm optimization	97.23	99.22	97.28	98.34	95.94	32.23
Particle swarm optimization	92.32	89.13	87.33	83.47	86.91	42.32

RETRACTED

## Data Availability

The data used to support the funding of this study are available from the corresponding author upon request.
